# Effect of Nursing in Operating Room Combined with Intraoperative Heat Preservation Intervention on Prevention of Incision Infection and Improvement of Hemodynamics in Patients with Anterior Cruciate Ligament Injury and Reconstruction under Knee Arthroscopy

This article has been retracted.

**DOI:** 10.1155/2022/2915157

**Published:** 2022-04-15

**Authors:** Jiao Dai, Yanan Li

**Affiliations:** ^1^Department of Operation, Wuhan Fourth Hospital (Puai Hospital Affiliated to Tongji Medical College of Huazhong University of Science and Technology), Wuhan, Hubei, China 430000; ^2^Department of Sport Medicine, Wuhan Fourth Hospital (Puai Hospital Affiliated to Tongji Medical College of Huazhong University of Science and Technology), Wuhan, Hubei, China 430000

## Abstract

**Objective:**

To explore the effect of nursing in operating room combined with intraoperative heat preservation intervention on preventing incision infection and improving hemodynamics in patients with anterior cruciate ligament (ACL) injury and reconstruction under knee arthroscopy.

**Methods:**

About 200 patients with knee arthroscopic ACL reconstruction in our hospital from January 2019 to July 2021 were enrolled. The patients were randomly assigned into two groups: the control group and the study group. The former group received nursing care in the operating room operating room and the latter group received nursing care in operating room combined with intraoperative heat preservation intervention. Nursing satisfaction, incidence of incision infection, knee joint VAS score, knee joint range of motion, knee joint Lysholm score, and hemodynamic indexes were compared.

**Results:**

First of all, we compared the nursing satisfaction, the study group was very satisfied in 78 cases, satisfactory in 20 cases, and general in 2 cases, and the satisfaction rate was 100.00%, while in the control group, 445 cases were very satisfied, 20 cases were satisfied, 15 cases were general, and 8 cases were dissatisfied. The satisfaction rate was 82.00%. The nursing satisfaction of the study group was higher compared to the control group (*P* < 0.05). Secondly, we compared the incidence of incision infection. The incidence of incision infection in the study group was lower compared to the control group (*P* < 0.05). With regard to the knee joint VAS score, the knee joint VAS score of the study group was lower compared to the control group at 2 weeks, 4 weeks, 8 weeks, and 12 weeks after operation (*P* < 0.05). In terms of the range of motion of the knee joint, the range of motion of the knee joint in the study group was higher compared to the control group at 2 weeks, 4 weeks, 8 weeks, and 12 weeks after operation (*P* < 0.05). Regarding the knee joint Lysholm score, the knee joint Lysholm score of the study group was higher compared to the control group at 2 weeks, 4 weeks, 8 weeks, and 12 weeks after operation (*P* < 0.05). Finally, we compared the hemodynamic indexes. Before nursing, there exhibited no significant difference (*P* > 0.05). During and after nursing, the indexes of HR and MAP in the study group fluctuated little (*P* < 0.05).

**Conclusion:**

During the perioperative period of patients with ACL injury and reconstruction under knee arthroscopy, standardized and necessary operating room combined with intraoperative thermal insulation intervention measures should be given, attention should be paid to the management of operating room, and intraoperative thermal insulation intervention should be strengthened. It includes preoperative visit, psychological nursing of patients, strict application of antibiotics before operation, monitoring of air quality in operating room, disinfection and sterilization of surgical instruments, shortening operation time, maintaining body temperature during operation, and paying attention to hand hygiene of medical staff. It plays a supervisory role in promoting the attention of medical staff to the prevention of wound infection, which is beneficial to the healing of surgical wounds of patients. It plays a positive role in enhancing hemodynamic indexes. Comprehensive nursing intervention on the risk factors of each link can effectively prevent postoperative wound infection and strengthen the prognosis and quality of life of patients.

## 1. Introduction

The operating room is a place to provide surgery and rescue for patients [1]. It is an important technical department of the hospital and an important place for surgery. Surgical site infection (SSI) is one of the most important complications of surgery, accounting for about 14.0% of all hospitalized patients infected with 16.0% [2]. Surgical wound infection is more common during the operation, there are many reasons, such as the patients' own reasons, and the vast majority of infections come from hospital infections [3]. Because there are many types of diseases in orthopedic patients, there are many kinds of orthopedic surgery, among which the more common types of surgery are reconstruction and repair surgery. Therefore, according to the different orthopedic surgery sites and causes, perioperative nursing methods are different, which is also a vital factor affecting surgical wound infection, and the quality of nursing in operating room determines the surgical effect to some extent [4]. In terms of the more open germ surgery, joint replacement surgery, spinal surgery, and closed fracture surgery are regarded as aseptic surgery and need to be implanted with prostheses and steel plates. Therefore, while strengthening preoperative preparation and postoperative prevention, nursing measures during the operation are also extremely important [5]. Postoperative wound infection causes delayed healing of incision and poor wound healing, which not only adversely affects the effect of operation but also prolongs the course of treatment of patients, affects the functional recovery of patients' limbs, and increases the economic and psychological burden of patients. It will adversely affect the quality of life of patients in the future; moreover, patients may bring about more serious complications and even face the risk of amputation. Severe wound infection can cause systemic infection and multiple organ dysfunctions, resulting in septic shock and even life-threatening. The smooth recovery of postoperative incision can enhance the patients' confidence in postoperative rehabilitation, promote their postoperative self-care and return to social life as soon as possible [6]. In order to effectively reduce the incidence of incision infection, it has been an important topic to strengthen and pay attention to the prevention and control of related infection. Through research and analysis, the factors causing incision infection come from many aspects, and the prevention of surgical wound infection is also the result of the joint action of many links, which is of great significance for the prevention of wound infection in the link of nursing intervention in operating room.

Anterior cruciate ligament (ACL) injury is a common knee injury disease in clinic. After ACL injury, the flexion, extension, and rotation of the knee joint will be unstable, which can lead to meniscus and articular cartilage injury. Early ACL reconstruction can prevent the secondary injury of the knee joint [7]. At present, arthroscopic minimally invasive surgery has been widely carried out in clinic, and compared with open surgery, arthroscopic minimally invasive surgery has the advantages of less trauma, less postoperative inflammatory reaction, rapid recovery, low incidence of infection, and clear surgical vision [7]. It has become the primary choice for the treatment of ACL injury. Although arthroscopic ACL injury and reconstruction are a minimally invasive operation, it is still invasive, and there are still symptoms such as swelling and pain at the early stage after operation. If the postoperative immobilization time is too long, it will lead to blood and lymphatic circulation stasis of the lower extremities, tissue edema, and reactive effusion of the knee joint, resulting in more morbid connective tissue [8]. Early postoperative safe and effective rehabilitation training has been widely recognized in clinic. Early rehabilitation training can not only promote the regression of knee joint swelling and reduce the incidence of knee joint adhesion, and isometric contraction training of quadriceps femoris and triceps calf can effectively reduce the incidence of disuse atrophy of muscles around knee joint and deep venous thrombosis of lower extremities [8]. However, the aggressive or high intensity of early postoperative rehabilitation training will aggravate the swelling and pain of the knee joint, make the patients lose confidence in the rehabilitation training, hinder the smooth progress of the rehabilitation training, and have a negative effect on the postoperative rehabilitation of the knee joint [9]. Therefore, how to reduce the knee joint inflammatory reaction after ACL reconstruction and eliminate the postoperative knee joint swelling and pain become more effectively. Some studies have pointed out that while perioperative nursing is carried out in operating room, intraoperative heat preservation intervention can not only effectively reduce the incidence of incision infection but also enhance hemodynamic indexes, which plays a positive role in postoperative rehabilitation [10]. Based on this, this study focuses on the effect of operating room nursing combined with intraoperative heat preservation intervention on preventing incision infection and promoting hemodynamics in patients with ACL injury and reconstruction under knee arthroscopy.

## 2. Patients and Methods

### 2.1. General Information

About 200 patients with knee arthroscopic ACL reconstruction in our hospital from January 2019 to July 2021 were enrolled. The patients were randomly assigned into two groups: the control group and the study group. The former group received nursing care in operating room, and the latter group received nursing care in operating room combined with intraoperative heat preservation intervention. This study was permitted by the Medical Ethics Association of our hospital, and all patients signed informed consent.

Diagnostic criteria were as follows: refer to “practical Orthopaedics” on the diagnostic criteria of ACL injury [8]: (1) history: patients have an obvious history of knee joint trauma: sprain, fall, and sports injury; (2) clinical manifestations: obvious swelling and pain of knee joint in the early stage of injury, obvious limitation of movement, no obvious swelling and pain of knee joint after old injury for more than 6 weeks, and instability of knee joint during daily life or exercise; (3) physical examination: front drawer test (+), Lachman test (+), axle shift test (+), and lever sign (+) [9]; and (4) auxiliary examination: X-ray: the anterior and lateral films of the knee joint usually show normal. If Segond fracture is found, it may indicate that there may be injury of ACL. MRI examination indicated that the continuity of ACL was interrupted, there was no tension in the ligament, and the ligament became thicker.

Inclusion criteria were as follows: (1) the patients who meet the above diagnostic criteria, (2) the patients whose age was from 18 to 50 years old, (3) simple ACL injury without other combined injuries, (4) arthroscopic single bundle ACL reconstruction operation in our hospital, (5) agree to give up other treatment measures that have nothing to do with this experiment, and (6) follow-up for at least 3 months.

Exclusion criteria were as follows: (1) less than 18 years old or more than 50 years old, (2) history of important vascular disease or nerve injury in lower extremities, (3) patients with serious medical diseases not suitable for operation, (4) patients with severe knee osteoarthritis, and (5) patients with mental illness who could not complete the postoperative rehabilitation plan as planned.

Termination, elimination, and shedding criteria were as follows: (1) shedding patients, (2) those who did not carry out or receive other related treatments according to the rehabilitation program, and (3) those with incomplete postoperative follow-up data caused by other reasons.

### 2.2. Treatment Methods

The control group received nursing care in operating room, and the specific measures were as follows: (1) preoperative nursing intervention is as follows: preoperative visit skin preparation nursing intervention: one day before operation, the instrument nurse visited the ward to have a comprehensive understanding of the patient's physical condition. Local disinfection of the operation site was carried out according to the patient's condition, and those who could not take a bath were locally disinfected with 2% chlorhexidine ethanol after bathing; the skin preparation condition of the patients was examined to reduce the possibility of incision infection. When the instrument nurses pick up the patients on the day of the operation, they should carefully check that the patients really need to remove the skin preparation in the hair area of the operation site and find the defects in time to correct them. Nursing intervention of visiting psychological status before operation: The nurses in the ward are required to actively communicate with the patients; explain the general procedure of the operation to the patients; help the patients to eliminate the psychology of tension, anxiety, and fear; and make the patients and their families fully understand the relevant knowledge of the operation. In addition, to create a warm and comfortable ward environment, it is necessary to explain the operations that affect the patient's psychological state, such as indwelling catheter and placing wound drainage tube, and tell its purpose, so that the patient can accept and match the operation during the operation. Nursing intervention to pick up patients on operation day: when picking up patients, instrument nurses communicate with doctors to understand the patient's condition, operation name, operation method and intraoperative posture, and special requirements; communicate with patients and listen to their opinions and requirements. Check the results of patients' crossmatching test, check whether there are hepatitis B, hepatitis C, AIDS, diabetes, and other conditions, formulate a nursing intervention plan in line with the patient's condition, and carry out timely and effective nursing intervention. (2) Intraoperative nursing intervention is as follows: hand surgical hand disinfection: the preparation of medical staff should strictly carry out aseptic technical operation to the medical staff participating in the operation and strictly do a good job of hand hygiene and disinfection. (3) postoperative nursing intervention is as follows: the protection of surgical incision: during the operation, a disposable incision protective film was used around the incision to protect the dressing around the incision from being dry, clean, and not contaminated. After the operation, the wound can be covered with disposable aseptic dressing, and the disposable negative pressure drainage box can be adopted for incision drainage. Keep the dressing intact and dry 48 hours after operation. When patients with wound infection are found, doctors should enhance their vigilance and awareness, register, and report to the hospital infection management department in time, and the hospital sensation department should assist in the cause analysis of wound infection, so as to promote the prevention awareness of medical staff and learn to prevent knowledge. Environmental hygiene of the ward is as follows: orthopaedics is the main surgical department of the hospital, pays attention to the environmental management of the ward, enhances the environmental hygiene of the ward, keeps the ward clean and quiet, arranges patients reasonably, and reduces attendants; wet cleaning is adopted in morning nursing and ventilated on time to reduce the dust in the air so as to reduce the pollution of bacteria and microorganisms, wipe the bedside table and bed unit, keep the ward bed unit and quilt clean, and improve the quality management of the environment inside and outside the ward and reduce the microbial pollution to the wound. Health education for discharged patients was routinely carried out, and patients were informed to review regularly at 1 month, 3 months, 6 months, and 12 months after operation, and telephone visits were carried out if necessary to understand the healing condition of discharged patients.

The study group received nursing care in operating room combined with intraoperative heat preservation intervention, and operating room nursing was the same as the control group. The specific measures of intraoperative heat preservation intervention were as follows: before the patient entered operating room, the temperature of operating room was controlled at 26°C, and after the operation began, the room temperature was adjusted to about 24°C. After entering operating room, the patient lay on the operation bed where the electric thermal insulation blanket was placed, and the thermal insulation blanket was adjusted to the appropriate temperature to cover the quilt to keep warm. The input liquid is heated by a liquid heating device in advance, so that the temperature of the liquid is slightly higher compared to the normal body temperature of the human body, but not more than 4°C, so as to avoid a series of body damage caused by the excessive temperature of liquid into the human body. The method of anesthesia was hard lumbar combined anesthesia, and the body temperature was measured by axillary temperature measurement. All operations were performed by the same group of doctors. The average body temperature was recorded before operation, after the beginning of anesthesia and during the operation. The average body temperature was measured, and the data were recorded per 15 min. The body temperature intervention group adjusted the temperature and infusion of the blanket according to the changes of the patient's body temperature during the operation and continued to use the blanket to resuscitate the anesthesia after operation to keep the patient's body temperature above 36°C. The routine treatment group did not use electric insulation blanket and could not warm up the infusion but only covered the patients with quilts.

### 2.3. Observation Index

#### 2.3.1. Satisfaction

After consulting the literature and experts' discussion, we designed patients' follow-up satisfaction, a total of 10 items, and recorded patients' satisfaction with follow-up management mode, health education, medical and nursing service, and appointment registration process [10]. It is assigned into four dimensions: very satisfied, satisfied, general, and dissatisfied: satisfaction rate = very satisfaction rate + satisfaction rate + general rate.

#### 2.3.2. Incidence of Incision Infection

Incision infection indicates that surgery which involves a cut (incision) in the skin can lead to a wound infection after surgery. The incidence of postoperative incision infection was calculated.

#### 2.3.3. Knee Joint Pain

The VAS score of knee pain in the two groups was recorded at 2 weeks, 4 weeks, 8 weeks, and 12 weeks after operation, which was a commonly used clinical pain evaluation method-visual analogue score [11]. The knee pain scores were recorded at 2 weeks, 4 weeks, 8 weeks, and 12 weeks after operation.

#### 2.3.4. Range of Motion of Knee Joint

The range of motion of the knee joint (ROM) is based on the maximum angle of the passive motion of the knee joint of the affected limb and is measured by a double-arm protractor [12]. The protractor is centered on the lateral condyle of the femur, one arm of the protractor is parallel to the femoral shaft, and the other arm is parallel to the tibial shaft. The angle between the two arms is the maximum angle of motion of the knee joint. The range of motion of the knee joint of the two groups was recorded at 2 weeks, 4 weeks, 8 weeks, and 12 weeks after operation.

#### 2.3.5. Knee Joint Function

Lysholm score is one of the international knee function scoring standards with high reliability and sensitivity [13]. The knee joint function Lysholm scores were followed up in the form of questionnaire at 2 weeks, 4 weeks, 8 weeks, and 12 weeks after operation.

#### 2.3.6. Hemodynamics

The heart rate and diastolic blood pressure were recorded before, during, and after nursing.

### 2.4. Statistical Analysis

The research data were statistically processed by SPSS 21.0 statistical software, the measurement data are expressed by ($\bar{x}\pm s$), and the counting data are expressed by *χ*^2^ test. If the measurement data conform to the normal distribution and the variance is uniform, two independent sample *t*-tests are employed for comparison. If the measurement data do not conform to the normal distribution or accord with the normal distribution but the variance is uneven, then using the nonparametric rank sum test. *P* < 0.05 is considered statistically significant while *P* < 0.01 is viewed as highly statistically significant in this study.

## 3. Results

### 3.1. Comparison of Nursing Satisfaction

First of all, we compared the nursing satisfaction. The study group was very satisfied in 78 cases, satisfactory in 20 cases, and general in 2 cases, and the satisfaction rate was 100.00%. The control group was very satisfied in 445 cases, satisfactory in 20 cases, general in 15 cases, and dissatisfied in 8 cases, and the satisfaction rate was 82.00%. In the control group, the age was 18-47 years old, with an average of (31.44 ± 3.64) years, including 48 males and 52 females, while in the study group, the age was 19-48 years old, with an average of (31.55 ± 3.77) years, including 46 males and 54 females. There was no statistical significance in the general data of the two groups. The nursing satisfaction in the study group was higher compared to the control group (*P* < 0.05). All the data results are indicated in Figure 1.

### 3.2. Incidence of Incision Infection

Secondly, we compared the incidence of incision infection. The incidence of incision infection in the study group was lower compared to the control group (*P* < 0.05). All the data results are indicated in Figure 2.

### 3.3. Comparison of VAS Score of Knee Joint

Thirdly, we compared the knee joint VAS score. The knee joint VAS score of the study group was lower compared to the control group at 2 weeks, 4 weeks, 8 weeks, and 12 weeks after operation (*P* < 0.01). All the data results are indicated in Table 1.

### 3.4. Comparison of Range of Motion of Knee Joint

Then, we compared the range of motion of the knee joint. The range of motion of the knee joint in the study group was higher compared to the control group at 2 weeks, 4 weeks, 8 weeks, and 12 weeks after operation (*P* < 0.01). All the data results are indicated in Table 2.

### 3.5. Knee Joint Lysholm Score Comparison

Next, we compared the knee joint Lysholm score. The knee joint Lysholm score of the study group was higher compared to the control group at 2 weeks, 4 weeks, 8 weeks, and 12 weeks after operation (*P* < 0.01). All the data results are indicated in Table 3.

### 3.6. Comparison of Hemodynamic Indexes

Finally, we compared the hemodynamic indexes. Before nursing, there exhibited no significant difference (*P* > 0.05). During and after nursing, the fluctuation of HR and MAP indexes in the study group was small (*P* < 0.01). All the data results are indicated in Table 4.

## 4. Discussion

ACL injury is one of the common knee joint injuries in clinic, accounting for about 80% of knee joint ligament injuries, mostly in sports injuries, and nonsports injuries account for 27.2% [14]. According to statistics, the annual incidence of ACL injury in the general population of the United States is 1 to 3 000, while the incidence of ACL injury in sports is even higher: 60/100000 for football players and 70/100000 for skiers [15]. The probability of ACL injury in female athletes is four times higher compared to men. The prevalence rate of ACL injury in active service athletes in China is 0.43%, with the improvement of living standards and health concepts. As more people participate in physical exercise, the probability of ACL injury increases [15]. ACL is an important anatomical structure in the knee joint, which starts from the anterior medial side of the tibial intercondylar eminence and ends at the back of the lateral wall of the intercondylar fossa. Most people think that ACL can be assigned into two bundles: anteromedial bundle (AMB) and posterolateral bundle (PLB) [16]. However, through anatomical observation, some scholars found that the imprinting of ACL at the end of the tibia was mostly close to the medial meniscus [17]. It was proposed that ACL could be assigned into AMB and posterior medial bundle (PMB), but there was no PLB. The study found that, when ACL was reconstructed by single bundle anatomy, it is confirmed from the other side that there may be no PLB in ACL. Other scholars have proposed that there is an intermediate beam of PLB stress transition between the two beams of ACL [18]. The external violence in ACL injuries can be assigned into contact injuries and noncontact injuries. Noncontact injuries account for 70-84% of all ACL injuries. Biomechanical studies have confirmed that ACL can limit excessive forward movement and internal rotation of the tibia and stabilize the flexion, extension, and rotation of the knee joint [19]. Therefore, if the knee joint activity exceeds the normal range of motion, ACL may be injured. For example, excessive internal rotation of the tibia caused by side rotation kicking in football and excessive valgus of the knee joint during a high-energy car accident or accidental fall may lead to ACL injury [20]. During the first visit of the patient, asking the cause of the injury, the existence of violence, and the injury action in detail can better judge whether the patient has ACL injury and the severity of the injury.

At present, there are three commonly used methods of ACL reconstruction: traditional isometric reconstruction, anatomical double-bundle reconstruction, and anatomical single-bundle reconstruction [21]. There are significant differences among the three surgical methods in the location of femoral tunnel. The theory of “isometric reconstruction” is the dominant idea of traditional single-bundle reconstruction. This theory holds that if the graft is always isometric in the flexion and extension of the knee joint, it can prevent the graft from breaking due to excessive load at a certain angle [22]. The study indicates that, within the range of 0-140° extension and flexion of the knee joint, it is an ideal isometric point near the “over-parietal position” behind the Blumensaat line, where the traditional single-bundle reconstruction of the femoral tunnel is located, while the anatomical double-bundle reconstruction of the femoral tunnel is located in the center of the attachment of the AMB and the posterior external bundle, respectively, and the anatomical single-bundle reconstruction of the femoral tunnel is located at the midpoint of the abovementioned two-center connection [23]. Biomechanical study found that the traditional single-bundle reconstruction can stabilize the flexion and extension of the knee joint but cannot well solve the stability of the rotation of the knee joint [23, 24]. Through biomechanical and clinical studies, foreign scholars have indicated that anatomical double-beam reconstruction is significantly better than traditional single-beam reconstruction in controlling rotational stability [25]. Through biomechanical study, it is found that single bundle anatomical reconstruction is better than traditional single bundle reconstruction in rotational stability, but there is no significant difference between anatomical double bundle reconstruction and anatomical double bundle reconstruction, and there are many problems in anatomical double bundle reconstruction. For example, the difficulty of operation, long operation time, and high cost of operation, not suitable for patients with small intercondylar fossa, etc., restricts its clinical application, while anatomical single-bundle reconstruction is relatively simple and more minimally invasive. It is suitable for most patients and is convenient to be carried out widely in clinic. An in-depth study of anatomical single-bundle reconstruction is conducive to the better recovery of knee joint function.

With the continuous improvement of people's living standards in our country, more patients with ACL injury hope that through surgical treatment, the knee joint function of the affected limb can be fully restored to the pre-injury level [26]. Minimally invasive arthroscopy has the advantages of clear vision, less trauma, mild postoperative inflammatory reaction, rapid recovery, and low incidence of infection, which brings hope of rehabilitation for patients with ACL injury [27]. Arthroscopic reconstruction of ACL has become the main treatment of ACL injury, but due to the lack of postoperative rehabilitation, postoperative complications such as adhesion of knee joint and muscle atrophy around knee joint occur. Affect the recovery of knee joint function, serious cases can lead to the loss of knee joint function [28]. SSI is one of the most serious postoperative complications so far, and the number of knee arthroscopic ACL reconstruction surgery is also increasing year by year [29]. It is an important topic for orthopaedic and operating room medical staff to prevent postoperative wound infection. Infection is a medical problem that perplexes human beings. How to prevent infection has always been a hot issue concerned by medical staff [30]. In nursing intervention in the prevention of knee arthroscopic ACL injury reconstruction surgical incision infection, many medical experts and scholars have done related research, to prevent wound infection, and the improvement of nursing intervention has made a great contribution [31, 32]. The human thermoregulatory system will control the core body temperature at about 37°C. When the internal core body temperature is out of the normal range, if the body's regulatory system cannot quickly restore the body temperature to normal, the environment in the body will lose balance and even worse, leading to the decline of organ function and a series of adverse events such as cardiocerebrovascular diseases. Perioperative hypothermia refers to mild hypothermia when the core temperature is lower than 36°C, and the body temperature is between 34 and 36°C [33]. Perioperative hypothermia is very common in surgery, with an incidence of 50% to 70% [34]. Its harm is also very obvious and can increase the incidence of deep wound infection, cardiac adverse events, and other complications but also increase the amount of blood loss of surgical patients [35]. In recent years, due to the increasingly mature development of surgical techniques, the incidence of perioperative hypothermia is getting higher. Meanwhile, due to more complications caused by hypothermia, perioperative hypothermia cannot be ignored. Intraoperative heat preservation intervention can effectively reduce the risk of hypothermia and enhance hemodynamic indexes to promote the smooth progress of the operation.

Conclusively, during the perioperative period of patients with ACL injury and reconstruction under knee arthroscopy, standardized and necessary operating room nursing combined with intraoperative thermal insulation intervention measures should be given, attention should be paid to operating room management, and intraoperative thermal insulation intervention should be strengthened. It includes preoperative visit, psychological nursing of patients, strict application of antibiotics before operation, monitoring of air quality in operating room, disinfection and sterilization of surgical instruments, shortening operation time, maintaining body temperature during operation, and paying attention to hand hygiene of medical staff. It plays a supervisory role in promoting the attention of medical staff to the prevention of wound infection, which is beneficial to the healing of surgical wounds of patients. It plays a positive role in enhancing hemodynamic indexes. Comprehensive nursing intervention on the risk factors of each link can effectively prevent postoperative wound infection and strengthen the prognosis and quality of life of patients.

## Figures and Tables

**Figure 1:** Comparison of nursing satisfaction between two groups. The green bar indicated control group, and the yellow bar indicated research group.

**Figure 2:** Incidence of incision of infection in two groups. The blue area indicated control group, and the orange area indicated research group.

**Table 1:** Comparison of knee joint VAS score between the two groups ($\bar{x}\pm s$, points).

Group	*N*	2 weeks after operation	4 weeks after operation	8 weeks after operation	12 weeks after operation
C group	100	5.79 ± 1.21	4.35 ± 1.23	3.17 ± 1.22	1.27 ± 0.66
R group	100	4.12 ± 0.67	3.11 ± 0.31	2.21 ± 0.64	0.56 ± 0.12
*t*		12.074	9.775	6.968	10.584
*P*		<0.01	<0.01	<0.01	<0.01

**Table 2:** Comparison of knee joint motion between the two groups ($\bar{x}\pm s$).

Group	*N*	2 weeks after operation	4 weeks after operation	8 weeks after operation	12 weeks after operation
C group	100	65.82 ± 2.31	78.38 ± 4.31	86.38 ± 4.77	114.69 ± 3.31
R group	100	70.91 ± 4.31	84.94 ± 4.65	98.83 ± 3.45	128.69 ± 5.66
*t*		10.408	10.346	21.148	21.351
*P*		<0.01	<0.01	<0.01	<0.01

**Table 3:** Comparison of knee joint Lysholm score between the two groups ($\bar{x}\pm s$, points).

Group	*N*	2 weeks after operation	4 weeks after operation	8 weeks after operation	12 weeks after operation
C group	100	73.49 ± 2.21	79.39 ± 3.31	84.81 ± 4.32	90.91 ± 5.31
R group	100	76.38 ± 2.24	84.35 ± 3.62	89.39 ± 1.25	94.39 ± 1.22
*t*		9.184	10.111	10.184	6.387
*P*		<0.01	<0.01	<0.01	<0.01

**Table 4:** Comparison of hemodynamic indexes between the two groups ($\bar{x}\pm s$).

Group	*N*	HR(time/min)			MAP(mmHg)		
		Before nursing	Nursing	After nursing	Before nursing	Nursing	After nursing
C group	100	80.93 ± 2.21	71.55 ± 1.56	89.93 ± 1.66	90.39 ± 3.31	99.24 ± 2.56	86.49 ± 3.34
R group	100	80.59 ± 2.34	80.49 ± 1.22	81.59 ± 2.21	90.59 ± 3.45	90.69 ± 3.31	90.59 ± 4.31
*t*		1.056	45.142	30.173	0.418	20.432	7.519
*P*		>0.05	<0.01	<0.01	>0.05	<0.01	<0.01

## Data Availability

No data were used to support this study.
